# Structure and mechanism of the essential two-component signal-transduction system WalKR in *Staphylococcus aureus*

This article has been retracted.

**DOI:** 10.1038/ncomms11000

**Published:** 2016-03-18

**Authors:** Quanjiang Ji, Peter J. Chen, Guangrong Qin, Xin Deng, Ziyang Hao, Zdzislaw Wawrzak, Won-Sik Yeo, Jenny Winjing Quang, Hoonsik Cho, Guan-Zheng Luo, Xiaocheng Weng, Qiancheng You, Chi-Hao Luan, Xiaojing Yang, Taeok Bae, Kunqian Yu, Hualiang Jiang, Chuan He

**Affiliations:** 1 Department of Chemistry, Department of Biochemistry and Molecular Biology, and Institute for Biophysical Dynamics, Howard Hughes Medical Institute, The University of Chicago, 929 East 57th Street, Chicago, Illinois 60637, USA; 2 State Key Laboratory of Drug Research, Drug Discovery and Design Center, Shanghai Institute of Materia Medica, Chinese Academy of Sciences, Shanghai 201203, China; 3 Shanghai Center for Bioinformation Technology, Shanghai Academy of Science and Technology, Shanghai 201203, China; 4 Synchrotron Research Center, LS-CAT, Northwestern University, Argonne, Illinois 60439, USA; 5 Indiana University School of Medicine-Northwest, Gary, Indiana 46408, USA; 6 High-Throughput Analysis Laboratory, Department of Molecular Biosciences, Center for Structural Genomics of Infectious Diseases, Northwestern University, Evanston, Illinois 60208, USA; 7 Department of Biochemistry and Molecular Biology, University of Chicago, 929 E 57th Street, Chicago, Illinois 60637, USA

## Abstract

Most low GC Gram-positive bacteria possess an essential *walKR* two-component system (TCS) for signal transduction involved in regulating cell wall homoeostasis. Despite the well-established intracellular regulatory mechanism, the role of this TCS in extracellular signal recognition and factors that modulate the activity of this TCS remain largely unknown. Here we identify the extracellular receptor of the kinase ‘WalK' (erWalK) as a key hub for bridging extracellular signal input and intracellular kinase activity modulation in *Staphylococcus aureus*. Characterization of the crystal structure of erWalK revealed a canonical Per-Arnt-Sim (PAS) domain for signal sensing. Single amino-acid mutation of potential signal-transduction residues resulted in severely impaired function of WalKR. A small molecule derived from structure-based virtual screening against erWalK is capable of selectively activating the *walKR* TCS. The molecular level characterization of erWalK will not only facilitate exploration of natural signal(s) but also provide a template for rational design of erWalK inhibitors.

## Abstract (web summary)

The WalKR signal transduction system is involved in extracellular signal recognition, but the details of this function are not well established. Here, the authors report the crystal structure of this two-component system alongside the characterisation of a small-molecule activator.

Signal transduction mediated by two-component systems (TCSs) is one of the primary strategies utilized by bacteria for adapting to changing environments. The sensor kinase, one major component of TCSs, plays a central role in extracellular stimuli recognition and intracellular autokinase activity modulation, leading to the transference of its phosphoryl group to the response regulator, another component of TCSs, for the downstream gene regulation in response to the signal(s)^1^,^2^.

*Staphylococcus aureus*, the leading cause of hospital- and community-acquired infections, has been the infectious disease with the highest mortality rate in the United States since 2007 (ref. 3) in large part because of the emergence of drug-resistant strains, such as methicillin-resistant and vancomycin-resistant *S. aureus*^4^. Besides antibiotic resistance, this human pathogen causes infections almost everywhere in the human body, consequently resulting in a variety of diseases ranging from minor skin infections to life-threatening diseases^5^,^6^. The versatility of this bacterium in pathogenesis is largely attributed to its capacity to coordinately express virulence factors according to changing environmental stimulus, mediated predominantly by its 16 TCSs (for example, *agrAC*, *saeRS* and *arlRS*) as well as key virulence regulators (for example, *sarA*, *mgrA* and *cymR*)^7^,^8^,^9^,^10^,^11^,^12^.

Among the 16 TCSs in *S. aureus*, WalKR (YycGF, VicKR and MicAB) is the only essential TCS involved in diverse cellular processes, including cell wall metabolism, virulence regulation, biofilm production, oxidative stress resistance and antibiotic resistance via direct or indirect regulation of autolysins, the *saeRS* TCS, haemolysins as well as other key virulence factors^13^,^14^,^15^,^16^. The sensor kinase of this TCS in *S. aureus*, WalK, possesses three functional domains including the intracellular kinase, the transmembrane helices as well as the extracellular receptor domain, the first two of which have been found to be conserved across the bacteria that contain this TCS. The other functional domain, the extracellular receptor domain (erWalK) is only present in the bacterial species (for example, *Bacillus subtilis*, *S. aureus*, *Enterococcus faecalis* and *Listeria monocytogenes*) in which this TCS is essential^14^. The response regulator of this TCS, WalR, is composed of two functional domains: the phosphorylation reception domain and the DNA-binding domain. Mutation of the phosphorylation reception residue Asp55 in WalR to a phosphomimetic residue Glu (WalRD55E) constitutively activates WalKR TCS, leading to enhanced expressions of a set of cell wall metabolism enzymes as well as numerous virulence factors^13^. Although extensive research has focused on elucidating the intracellular regulatory mechanism of WalKR TCS^13^,^15^,^16^,^17^,^18^,^19^ and past studies have explored the role of the transmembrane helices of *B. subtilis* WalK in modulating kinase activity through interactions with auxiliary proteins YycH and YycI^20^,^21^, little is known about the role and mechanism of erWalK in signal recognition and consequent kinase activity modulation.

Here we report the crystal structure of erWalK, revealing a canonical Per-Arnt-Sim (PAS) domain for signal recognition. We demonstrate the key role of erWalK in potential signal recognition and kinase activity modulation. Because of the extracellular nature of this domain, small molecules can target erWalK directly from the outside in order to modulate its function and/or treat *S. aureus* infection. Through structure-based virtual screening, we discovered a small molecule, which activates WalKR TCS via targeting erWalK, thus demonstrating the feasibility of this strategy.

## Results

### Structural characterization of erWalK

The sequence of the extracellular receptor of the sensor kinase WalK indicates a PAS domain known for signal detection and transduction^20^. The failure of our previous attempts to deplete the entire extracellular receptor domain (amino acids: T34-Q182) in *S. aureus* has prevented our detailed understanding of the role of this domain in signal transduction. We sought to determine the crystal structure of erWalK in order to probe its function biochemically and genetically based on the structural information.

To facilitate the crystallization of erWalK, seven distinct constructs harbouring different truncations of the extracellular domain between the two transmembrane helices were cloned, expressed and screened (Supplementary Table 1). One construct containing the entire extracellular receptor region erWalK6 was successfully crystallized with the crystals diffracting to 2.1 Å resolution (Supplementary Table 1). However, the highly anisotropic property of the diffraction data prevented further data processing, which was likely ascribed to the presence of imperfect crystals formed by a mixture of different forms (monomer and dimer) of erWalK6 protein (Supplementary Fig. 1a). Further screening of single amino-acid mutants of erWalK6 yielded the construct erWalK6R86M (Arg86 was mutated to Met) that not only exhibited a single peak in size exclusion chromatography analysis (R86M in Supplementary Fig. 1a) but also was crystallized with the crystals diffracting to 1.7 Å resolution. The diffraction data could be processed and the structure was solved by using the seleno-methionine-labelled erWalK6R86M in phase determination (Table 1).

The crystal structure of erWalKR86M revealed that there are two protein molecules in the asymmetric unit that appear to form a tightly packed dimer (Fig. 1a). The biological relevance of this dimer is unknown; the erWalK686M protein does not form dimer in solution and the dimer is barely found in the wild-type protein when present in high concentrations (Supplementary Fig. 1a). Each monomer adopts a canonical PAS domain fold with the presence of five central antiparallel β-strands in a topological order of 2-1-5-4-3 (Fig. 1a,b)^22^. The ends of each monomer are two long helices, directly linking to the transmembrane helices, possibly bridging signal transduction from the extracellular receptor domain to the intracellular kinase domain. The mutation site MSE86 is located in the loop region between the second α-helix and the first β-strand with the side chain of MSE86 facing outwards (Supplementary Fig. 1b). Therefore, this mutation is less likely to change the overall structure of the protein, but may contribute to the crystallization.

PAS domain proteins often share a high degree of similarity in the overall tertiary structure, despite the relatively low sequence identity^23^. We therefore overlaid the erWalK PAS domain with a well-characterized DcuS PAS domain (root mean square deviation (r.m.s.d.) of 2.74 Å) (ref. 24) to probe the potential signal-recognition mode of erWalK. Four residues of D119, Y165, V149 and K138, residing in the core of erWalK PAS domain, were predicted to engage in signal transduction (Fig. 1c and Supplementary Fig. 1c). Further sequence alignment of *S. aureus* erWalK with three homologous erWalK proteins from three distinct low GC content Gram-positive bacteria revealed a high-degree conservation of D119, Y165 and V149 (in some cases, V149 is substituted by Ile), despite a relatively low overall incidence of sequence conservation (Supplementary Fig. 2a).

### Mutation of D119 or V149 to Ala dramatically impaired the function of WalKR

To genetically investigate the role of erWalK in WalKR-mediated signal transduction, we sought to create single amino acid substitutions of the aforementioned amino-acid residues by pKOR1-mediated allelic replacement^25^; we envisioned that such mutants might be viable and could reveal functional phenotypes associated with erWalK as the entire receptor itself may be essential in *S. aureus*. We successfully created two erWalK mutants containing single amino-acid substitutions of D119A and V149A (Asp119 and Val149 were mutated to Ala), respectively.

The WalKR TCS is known to regulate the cell wall structure with the depletion of this TCS leading to increased resistance to lysostaphin-induced lysis^15^. Therefore, we performed a lysostaphin-induced lysis assay to examine the function of the erWalK mutants. As shown in Fig. 2a, mutation of either D119 or V149 to Ala significantly retarded lysostaphin-induced lysis process, which could be restored by introducing a single-copy plasmid p-*walKR* containing the wild-type *walKR* gene. It is worth noting that mutation of either D119 or V149 to Ala in erWalK did not result in defects in cell growth, but in fact marginally accelerated cell growth (Supplementary Fig. 2b).

Because many major *S. aureus* virulence factors including hemolysin genes *hla*, *hlb* and *hlgABC* were reported to be positively regulated by *walKR* via the activation of *saeSR* TCS (ref. 13), we employed a sheep blood plate assay to further study the *walK* mutant strains. As shown in Fig. 2b, while both mutations exhibited almost fully abolished hemolysin production, the phenotype could be restored by introducing a single copy of *walKR*. The decreased expressions of hemolysin genes (*hla* and *hlgC*) in the mutants were confirmed by qRT-PCR (quantitative real-time PCR with reverse transcription) (Supplementary Fig. 3a). In addition, the central role of these residues in WalKR-mediated signal transduction was further shown by the reduced biofilm production of the mutant strains compared with the wild-type Newman strain (Fig. 2c) as well as decreased survival of *S. aureus* inside mice using a murine abscess model of infection (Fig. 2d); WalKR TCS has been shown to affect biofilm production and the pathogenesis of *S.aureus*^13^. Together, all these observations lead to the conclusion that D119 and V149 of erWalK play important roles in the signal-recognition core of WalKR.

Single amino-acid mutation may trigger protein misfolding and aggregation^26^,^27^. To exclude the possibility that the observed phenotypes of the D119A and V149A mutants result from misfolding or aggregation of erWalK after mutation, we cloned, expressed and purified three proteins erWalKR86M, erWalKR86MD119A and erWalKR86MV149A from *Escherichia coli* and subjected these recombinant proteins to size exclusion chromatography analysis. As shown in Supplementary Fig. 3b, erWalKR86MD119A and erWalKR86MV149A share a similar elution volume as that of erWalKR86M, with only a tiny amount found in the aggregates region (elution volume <45 ml), thus excluding the possibility that the mutation of D119 or V149 to Ala leads to protein aggregation.

Because we were unable to make the Y165A mutant, we made the Y165F mutant to study the role of Y165 in signal transduction. As shown in Supplementary Fig. 3c,d, mutation of Y165 to phenylalanine slightly reduced the lysostaphin-induced lysis activity, and slightly affected the expression of the hemolysin gene *hlgC*.

Despite the well-characterized role of WalKR TCS in affecting cell morphology in *Streptococcus pneumoniae*^28^, the impact of this TCS on cell morphology and wall property remains unknown in *S. aureus*, mostly because of the lack of a proper *walKR* mutant strain. We therefore employed transmission electron microscopy to image the *walK* D119A and V149A mutant strains and compared them with the wild-type strain. Interestingly, dramatically defective cell morphology (altered cell shape and asymmetric daughter cells) as well as slightly altered cell shape, were observed in the D119A (Fig. 3) and V149A (Supplementary Fig. 4a) mutants, respectively, revealing the critical role of WalKR TCS in the regulation of cell morphology in *S. aureus*. However, the cell wall thickness was not affected by the mutations (Supplementary Fig. 4b).

### Global transcription changes in the D119A and V149A mutants

To further understand the role of D119 and V149 in WalKR-dependent regulation in *S. aureus*, we performed RNA-seq analysis to compare the transcriptomes of D119A and V149A mutants with that of the Newman wild-type strain. In total, 190 (Supplementary Table 2) and 123 (Supplementary Table 3) genes with a greater than two-fold decrease in transcription levels were observed in the D119A and V149A mutants, respectively, as compared with the wild-type strain, with 111 genes observed for both mutants (Fig. 4a). On the other hand, 293 (Supplementary Table 4) and 180 (Supplementary Table 5) genes with a greater than two-fold increase in their transcription levels were found in the D119A and V149A mutants, respectively, as compared with the wild-type strain, with 174 genes obtained in both mutants (Supplementary Fig. 5). The more conservative change of the V149A mutation as compared with the D119A mutation may contribute to the observation of more differentially expressed genes in the D119A mutant strain as compared with the V149A mutant strain.

Moreover, genes differentially expressed in the D119A mutant were found to play diverse roles in cellular processes, including cell wall metabolism, pathogenesis, regulatory pathway, metabolism, transporter, cell wall synthesis and transcription (Fig. 4b). Notably, a majority of the downregulated genes are involved in cell wall metabolism (*lytM*, *NWMN_0150*, *NWMN_2203* and *NWMN_2469*), pathogenesis (*coa*, *chp*, *hla* and *hlgABC* and so on), and the regulatory pathway (*saeSR*) in the D119A mutant, which agrees with microarray results of upregulated genes in a constitutively active *walR* mutant *walRD55E* (Fig. 4c)^13^. Besides the downregulated genes involved in cell wall metabolism and pathogenesis in both mutants, a striking observation is the upregulation of a capsular polysaccharide synthesis gene cluster (from *capA* to *capO*, Supplementary Tables 4 and 5) involved in resistance to the human innate immune system^29^ as well as cell wall synthesis genes (*murA* and *NWMN_2463*, Supplementary Tables 4 and 5) that have not been connected to the WalKR system before.

### A small molecule targeting erWalK activated the WalKR TCS

WalKR, as an essential TCS in *S. aureus*, has attracted increasing attention as a potential anti-infection target^30^,^31^. Previous attempts to target this TCS mostly focused on developing inhibitors against the intracellular kinase domain, such as the WalK kinase inhibitor waldiomycin^31^. While most sensor kinases share similar tertiary structures of their histidine kinase domains for ATP binding, their extracellular receptor domains often possess distinct signal-binding cores to serve roles in signal recognition, which therefore render the receptor domains as potential anti-infection targets with high specificity. In addition, targeting erWalK avoids potential delivery issues because of its extracellular localization. With the structural information in hand, we employed a structure-based virtual screening^32^, a widely utilized computational strategy in small-molecule screening, to identify small molecules that may bind erWalK and modulate the WalKR TCS. A total of more than 200,000 small molecules from SPECS database were screened and filtered, yielding 68 compounds that may bind erWalK.

Using a thermal shift assay^33^, we examined interactions between erWalK and the small molecules identified from the structure-based virtual screening. One small molecule 2, 4-dihydroxybenzophenone (DHBP), is capable of stabilizing erWalK as a titration of erWalK with increasing amounts of DHBP led to an elevated melting temperature with a maximum increase of 2.9 °C (Fig. 5a), indicating a direct interaction of DHBP with erWalK. The interaction between DHBP and erWalK was further confirmed by the surface plasmon resonance (SPR) analysis (Supplementary Fig. 6a). We next applied the lysostaphin-induced lysis assay to probe the interaction between DHBP and erWalK in life cells. As shown in Fig. 5b, DHBP at a concentration of 75 μM is capable of significantly accelerating the lysis process in the Newman wild-type strain (black dash curve in Fig. 5b), but not in the D119A mutant strain (purple dash curve in Fig. 5b) in which the lysis process remains the same with or without DHBP. This result confirmed the binding of DHBP to erWalK and indicated the involvement of residue D119 in DHBP binding. The lysis process could be slightly accelerated by DHBP in the V149A mutant strain (blue dash curve in Fig. 5b), but the extent is much less compared with that in the wild-type strain. It is worth noting that the supplementation of 75 μM DHBP did not affect the growth of the Newman wild-type strain (Supplementary Fig. 6b). The role of DHBP in activating WalKR TCS was further shown by significantly increased biofilm production. The supplementation of 75 μM DHBP increased biofilm production by ∼1.8-fold in the Newman wild-type strain (Supplementary Fig. 6c).

To gain insights into the binding of DHBP to erWalK, we performed computational modelling, which revealed that DHBP binding may trigger a conformational change of the sensor domain. In the ligand-free erWalK conformation, the binding pocket is filled by side chains of E91, R93, V149, Y165 and E167 (Supplementary Fig. 7a). The salt bridges between E91 and R93, K138 and E167, and the hydrogen bonds between Y165 and E167, Y140 and E167 stabilize the ligand-free conformation (Supplementary Fig. 7a). Because the ligand-binding core in the ligand-free structure of erWalK is occupied by the side chain of Y165, the side chain of Y165 has to rotate out to generate a cavity for DHBP binding (Supplementary Fig. 7b,c). After rotation, the packing between the α-helix, where D119 locates, and the β-sheet, where V149 locates, may contribute to the stabilization of the side chain of Y165 (Supplementary Fig. 7d,e). The carboxyl group of D119 forms hydrogen bonds with the amino groups of S121 and V122 (Supplementary Fig. 7b,c). Mutation of D119 to alanine may reduce the stability of the α-helix. In addition, mutation of D119 to alanine may enlarge the cavity where the side chain of Y165 locates, therefore destabilizing the ligand-bound structure of erWalK. The conformational change (Supplementary Fig. 7f) occurred in the DHBP-binding region triggered by DHBP binding likely transfers to the intracellular kinase domain to modulate the kinase activity.

### DHBP treatment triggered profound transcriptional changes

To further investigate the role of DHBP as an activator of WalKR TCS, we performed RNA-seq to globally analyse transcriptome changes caused by DHBP supplementation in the Newman wild-type strain. In total, 145 genes were differentially expressed when the wild-type strain was treated with 50 μM DHBP, among which 95 genes were upregulated (Supplementary Table 6) and 50 genes were downregulated (Supplementary Table 7). Because WalKR TCS plays a positive regulatory role in the expression of cell wall metabolism and pathogenesis genes, we overlapped the 95 genes that were upregulated by the DHBP treatment with the downregulated genes (190) observed in the D119A mutant as compared with the wild-type. We found 41 overlapping genes (Fig. 6a). The remaining 54 genes were only present in the transcriptome profiling triggered by DHBP (Fig. 6a), suggesting that DHBP may also affect other pathways. Notably, a majority of upregulated genes upon DHBP treatment are involved in cell wall metabolism and pathogenesis, including *NWMN_2469*, *coa*, *fnbB*, *hlgA*, *NWMN_0757*, *NWMN_1075*, *set11nm*, *set7nm* and *set8nm*, which were found to be downregulated in the D119A mutant as compared with the wild-type strain (Figs 6b and 4c). In addition, four capsular polysaccharide synthesis genes, namely *capA*, *capB*, *capC* and *capD* that were upregulated in the D119A mutant were downregulated with the DHBP treatment in the Newman wild-type strain (Supplementary Table 7). Together, the transcriptome profiling supports the role of DHBP in activating WalKR TCS.

## Discussion

Despite the essential role of WalKR TCS in *S. aureus* survival^13^,^14^,^15^, the extracellular signalling domain has never been structurally characterized with little known about factors that modulate the activity of this TCS. Here we present the crystal structure of this key extracellular receptor domain of the sensor kinase WalK (erWalK). Our subsequent genetic studies designed based on the structure confirmed that erWalK functions as a key hub in bridging extracellular signal input and intracellular kinase modulation. Mutations of potential signal-transduction residues in erWalK led to attenuated WalKR TCS activity, whereas targeting erWalK by a synthetic molecule resulted in activation of this TCS.

Besides possessing the extracellular PAS domain, *S. aureus* WalK also contains a relatively conserved intracellular PAS domain (amino acids: H271-V366); the structure of a homologous protein in *Streptococcus mutans* has been determined^34^. Tertiary structure comparison of these two PAS domains reveals very distinct ligand-binding cores with r.m.s.d. of 6.37 Å (Supplementary Fig. 8), suggesting the presence of different types of extracellular and intracellular WalK signals. Notably, despite the relatively low overall sequence identity of the extracellular cellular PAS domain of WalK, the high-degree conservation of the potential signal-binding residues suggests the presence of conserved signal(s) shared by the bacteria that possess the extracellular PAS domain (Supplementary Fig. 2a).

In summary, we report the crystal structure of an erWalK in *S. aureus*, and demonstrated the critical roles of erWalK in signal recognition and intracellular kinase activity modulation. Several residues were identified as potential signal-transduction residues. Mutations of these residues to Ala led to functionally impaired WalKR TCS; the mutant strains showed dramatically attenuated virulence in a mouse model and reduced pathogenesis in other assays. Because erWalK is critical for WalKR TCS activity and is extracellular, it presents an ideal target for treating *S. aureus* infection with potential small molecules that can directly target this domain from the outside. Indeed, we discovered a small-molecule DHBP by structure-based virtual screening, which is capable of activating WalKR TCS through targeting erWalK. When both agonists and antagonists bind to the same protein pocket, they often share high structural similarity. Different modulation mechanisms can be achieved by introducing different functional groups in small molecules^35^,^36^. The agonist DHBP that is suggested to bind to erWalK in the present study may provide a scaffold structure for designing and synthesizing new agents with higher affinity. The interactions critical to the tuning of WalKR activity can also help future design of erWalK inhibitors.

## Methods

### Bacterial strains, primers, plasmids and growth conditions

All the bacterial strains, plasmids and primers used in this study are listed in Supplementary Tables 8 and 9. *E. coli* strains were cultured in Luria-Bertani broth (LB). *S. aureus* strains were cultured in tryptic soy broth (TSB). Heart infusion broth supplemented with 5 mM CaCl_2_ was used for transduction procedures for *S. aureus*. When necessary, antibiotics were added at the following concentrations: ampicillin, 100 μg ml^−1^; and chloramphenicol, 10 μg ml^−1^. Vector pMCSG7 was used for recombinant protein expression. *E. coli*–*S. aureus* shuttle vector pCL55 was utilized for complementation. *E. coli*–*S. aureus* shuttle vector pKOR1 was used for single-nucleotide mutation in *S. aureus* genome.

### Protein expression and purification

The DNA fragments of seven erWalK constructs were PCR amplified from *S. aureu*s Newman genomic DNA and they were cloned into a protein expression vector pMCSG7 by the ligation independent cloning method^37^. One of the resulting plasmids pMCSG7-His-erWalK6 was mutated by the QuickChange II site-directed mutagenesis method (Agilent Technologies) to make the pMCSG7-His-erWalK6R86M and pMCSG7-His-erWalK6I58M plasmids. These plasmids were then transformed individually into an *E. coli* BL-21 strain for recombinant protein expressions.

To express the recombinant proteins, the BL-21 strains carrying the aforementioned plasmids were grown in LB medium to an OD_600_ of ∼0.6 at 37 °C. The cells were then cooled down to 16 °C and supplemented with 1 mM isopropyl β-D-1-thiogalactopyranoside (IPTG). The induced cells were further grown at 16 °C for 18 h. After collection, the cells were frozen at −80 °C. To express the seleno-methionine-labelled protein, a 10 ml overnight culture of the BL-21 strain containing pMCSG7-His-erWalK6R86M was collected and resuspended into 1 L of M9 minimal media (200 ml 5xM9 salts (64 g Na_2_HPO_4_-7H_2_O; 15 g KH_2_PO_4_; 2.5 g NaCl; and 5 g NH_4_Cl to 1 l H_2_O); 20 ml 20% glucose; 1 ml 0.1 M CaCl_2_; 2 ml 1 M MgSO_4_; and 0.1 ml 0.5% thiamine to 800 ml H_2_O). After the cells were grown at 37 °C to an OD_600_ of ∼0.6, they were supplemented with an amino-acid mixture (100 mg lysine (hydrochloride), 100 mg threonine, 100 mg phenylalanine, 50 mg leucine, 50 mg isoleucine, 50 mg valine and 60 mg seleno-methionine). The cells were further grown at 37 °C for 15 min before addition of 1 mM IPTG. The induced cells were then grown overnight at 37 °C before collection and freezing at −80 °C.

To purify the recombinant proteins, the cells were resuspended in buffer A (500 mM NaCl, 10 mM Tris-HCl, pH 7.5, 5% glycerol and 1 mM DTT) and lysed by sonication. The supernatent of the lysed cells were loaded onto Ni-NTA columns (Qiagen) individually and the proteins were purified by following manufactures' instructions. The proteins were further purified by a gel-filtration column (superdex 75, GE Healthcare) with a gel-filtration buffer (100 mM NaCl, 10 mM Tris-HCl, pH 7.5 and 1 mM DTT).

### Protein crystallization

Gel filtration-purified proteins (20 mg each) were mixed with the TEV protease (1 mg ml^−1^, 500 μl) individually and incubated overnight at 4 °C to cleave their polyhistidine tags. The mixture was then loaded onto a Ni-NTA column and the flow-through fraction was collected and concentrated to 2 ml before being purified by gel-filtration in the gel-filtration buffer. Each of the purified proteins was concentrated to 1.35 mM and used to screen for 800 conditions for crystallization. The seleno-methionine-labelled erWalK6R86M protein was crystallized in a buffer containing 0.2 M ammonium citrate dibasic, 20% w/v polyethylene glycol 3350 and pH 5.1 by sitting-drop method. The crystals were cryoprotected with a reservoir solution containing 22% glycerol and were frozen in liquid N_2_.

### Data collection, structure determination and refinement

The seleno-methionine-labelled erWalK6R86M crystal data was collected at the macromolecular crystallography beamline 21-ID-G at Advanced Photo Source, Argonne National Laboratory. The data was processed by HKL2000 (ref. 38) and the structure was solved by using single-wavelength anomalous dispersion (each monomer contains one molecule seleno-methionine at its 86 position). The phase was calculated by SOLVE and the density was modified by RESOLVE in PHENIX (ref. 39). The first round model was built by AutoBuild in PHENIX (ref. 39) and further improved by Coot and co-workers^40^ and REFMAC5 in the CCP4i software suit^41^. The final structure was validated by Procheck in the CCP4i software suit^41^ and visualized by PyMOL (http://www.pymol.org/).

### Construction of V149A, D119A and Y165A mutants

The allelic exchange plasmid pKOR1 was utilized to mutate a single amino acid of erWalK in *S. aureus*. In brief, the DNA fragment covering the *walKR* gene was PCR amplified from *S. aureus* Newman genomic DNA by primers WalKattB1/2 and further cloned into pKOR1 by the Gateway BP cloning method, resulting in a plasmid pKOR1∷*walK*. The mutation was performed by the QuickChange II site-directed mutagenesis (Agilent Technologies) method with the plasmid pKOR1∷*walK* as the template. The mutated plasmid was first transformed into RN4220 by electroporation and then into Newman wild-type strain by phage 85. Integration of the plasmid was performed by growing cells at the non-permissive condition (42 °C) with the presence of 10 μg ml^−1^ chloramphenicol and then excision of the plasmid was performed by growing cells at the permissive condition (30 °C) with the supplementation of 1 μg ml^−1^ anhydrotetracycline. The mutation in *S. aureus* genome was verified by sequencing the PCR product of *erwalK* amplified from the mutants' genome.

### Complementation of V149A and D119A mutants

The *E. coli*–*S. aureus* shuttle vector pCL55 was utilized for complementation. In brief, the ORF along with the promoter of *walKR* were PCR amplified from *S. aureus* Newman genomic DNA by primers WalKR_pCL55F/R. The PCR product was further cloned into the pCL55 vector. The resulting plasmid was first transformed into RN4220 by electroporation and then into the V149A and D119A mutants by phage 85.

### Lysostaphin-induced lysis assay

The overnight cultures of different *S. aureus* strains were 1:100 diluted into fresh TSB with the supplementation of 75 μM DHBP when indicated. The cells were grown to an OD_600_ of 1.2–1.7 before harvesting (10 min, 5,400*g*). The harvested cells were resuspended in PBS to make bacterial suspensions with an OD_600_ of∼1, which were further supplemented with 200 ng ml^−1^ lysostaphin. The suspensions were incubated at 37 °C with aeration and OD_600_ was monitored at different time points. The measured OD_600_ was normalized by dividing the initial OD_600_ for presentation.

### Blood plate assay

An amount of 1 μl overnight cultures of different *S. aureus* strains grown in TSB were loaded onto a sheep blood plate (TEKNOVA). The plate was incubated at 37 °C for 24 h and further stored at 4 °C for 24 h before being photographed.

### Quantitative real-time PCR

Cells were grown overnight at 37 °C in TSB. They were 1:100 diluted into fresh TSB and grown to the mid-log phase (OD600∼0.6). Cells were harvested by centrifugation and lysed by a beat beater. RNAs were extracted by the RNeasy Mini Kit (Qiagen) with DNase I treatment. qRT-PCR was performed by utilizing the SuperScript III Platinum SYBR Green One-Step qRT-PCR Kit (invitrogen) with 16 S rRNA as the internal control.

### Biofilm production assay

The overnight cultures of different *S. aureus* strains were 1:100 diluted into fresh TSB containing 0.5% glucose and 3% NaCl with the supplementation of 75 μM DHBP when indicated. After the cultures were grown in a polystyrene 96-well plate at 37 °C for 24 h, the wells were washed with PBS, dried and stained with 0.1% crystal violet for 20 min. The wells were further washed with PBS and air dried. Ethanol-acetone (80:20) was utilized for eluting the stained biomass, which was quantified by UV–vis at 595 nm.

### Murine infection and abscess formation

The Newman wild-type strain, V149A and D119A mutants were grown at 37 °C overnight in TSB. Cell cultures were then 1:100 diluted into fresh medium and incubated at 37 °C for 2.5 h until the cultures reached to an OD_600_ of ∼1.0. Bacteria were collected by centrifugation, washed and suspended in PBS buffer. A total of 100 μl of bacterial suspension (1 × 10^7^ colony forming units (CFU)) was administered intravenously via retro-orbital injection into each of 10 6-week-old BALB/c mice. Five days after injection, the animals were killed by CO_2_ asphyxiation and organs were removed. The organs were homogenized in 1 ml of PBS and dilutions of the homogenates were plated on TSA to calculate the number of bacteria. The experiment was carried out in strict accordance with the recommendations in the Guide for the Care and Use of Laboratory Animals of the National Institutes of Health. The protocol was approved by the Institutional Animal Care and Use Committee of the University of Chicago. All surgery was performed under sodium pentobarbital anaesthesia, and all efforts were made to minimize suffering.

### Transmission electron microscopy

The Newman wild-type strain, V149A, and D119A mutants were grown at 37 °C overnight in TSB. Cell cultures were then 1:100 diluted into a fresh medium supplemented with 75 μM DHBP when indicated and incubated at 37 °C for 2 h until the cultures reached to an OD_600_ of ∼0.6. Bacteria were collected by centrifugation and washed with PBS. The bacterial samples were fixed with a fixative (2% glutaraldehyde and paraformaldehyde in 0.1 M sodium cacodylate buffer) for 2 h, which were further washed with 0.1 M sodium cacodylate buffer (3 × 5 min). The cells were post fixed with 1% osmium tetroxide in 0.1 M sodium cacodylate buffer for 60 min. The cells were then washed with sodium cacodylate buffer (2 × 5 min) and rinsed with maleate buffer (1 × 5 min). The cells were further fixed by 1% uranyl acetate in maleate buffer for 60 min and washed with maleate buffer (3 × 5 min). The cells were dehydrated by the following steps: 25% ethanol (2 × 5 min); 50% ethanol (2 × 5 min); 70% ethanol (2 × 5 min); 95% ethanol (2 × 5 min); 100% ethanol (3 × 15 min); and 100% propylene oxide (3 × 15 min). The cells were then infiltrated by the following steps: 2:1 propylene oxide:spurr resin (2 × 30 min); 1:1 propylene oxide:spurr resin (2 × 30 min and overnight); 100% spurr resin (6 × 60 min). The spurr was polymerized with embedded cells in 60 °C oven for 1–2 days and then 90 nm sections were cut by Reichert-Jung Ultracut E. The samples were further stained with uranyl acetate and lead citrate and imaged under 300 KV at FEI Tecnai F30 with Gatan CCD digital micrograph.

### RNA-seq and data analysis

The Newman wild-type strain, V149A, and D119A mutants were grown at 37 °C overnight in TSB. Cell cultures were then 1:100 diluted into fresh TSB supplemented with 50 μM DHBP when indicated and incubated at 37 °C for 2 h until the cultures reached an OD_600_ of∼0.6. Bacteria were collected by centrifugation and washed with PBS. The cells were lysed by a bead beater and the total RNA was extracted by using an RNeasy minikit (Qiagen) with DNase I treatment step. The rRNA was removed by a MICROBExpress kit (Ambion) and the remaining RNA was utilized to construct the cDNA library by a TruSeq RNA sample prep kit (Illumina). The library was sequenced by next-generation sequencing (HiSeq 2000 (Illumina)). The sequencing reads were mapped to the *S. aureus* Newman strain genome by TopHat (version 2.0.0) with two mismatches allowed^42^. Cutffdiff software (version 2.0.0) was used to perform gene differential expression analysis^43^. Genes were annotated by BLAST and the Database for Annotation, Visualization and Integrated Discovery (DAVID) v6.7 (http://david.abcc.ncifcrf.gov). The experiments were performed in duplicate.

### Structure-based virtual screening

Since ligand binding in PAS domain proteins will often trigger significant conformational changes, the crystal structure of citrate-bound periplasmic domain of the sensor histidine kinase CitA (PDB id: 2J80)^44^ was used as the template to build the ligand-bound structure of erWalK. The model was then built using the online server of Swiss Modeler^45^,^46^ and refined by Discovery Studio2.5 using the force field of Charmm.

SPECS database that contains more than 200,000 compounds was used for virtual screening against the refined ligand-bound erWalK model. Glide in maestro package was used for virtual screening. After filtering out the small molecules with molecular weight larger than 400, the remaining ligands were then prepared using the application of LigPrep in maestro. OPLS_2005 force field was applied to all the ligands. Possible states were generated using Epik at target pH 7.0. Stereoisomers were computed retaining specified chirality. Conformation with the lowest energy ring conformation was generated. Target file from the refined modelled ligand-bound form of erWalk was prepared using the workflow of Protein Preparation Wizard in maestro. Hydrogen atoms were added and the H-bonds were optimized. Energy minimization was then performed to refine improper atoms using OPLS2005 force field. Receptor grid generating was then performed using Glide. The ligand site at 2J80 was used for the ligand-bound form of target. A grid box centred on the ligand-binding site with a length of 8 Å was set for grid generating. The ligands were docked to the receptor with standard precision. Dock flexible parameters were chosen in the process of docking. The resulting docked poses were then sorted by their docking scores. A total of 1,309 small molecules with Docking Score SP_score<-7 were used for further analysis. To obtain a structural diversity of small molecules, Discovery Studio was used to cluster the 1,309 small molecules into 80 clusters using the predefined properties. The PAINS compounds were then filtered^47^, yielding 68 compounds that potentially bind to erWalK.

### Fluorescence thermal shift assay

The fluorescence thermal shift assay was performed in a 384-well PCR plate with an assay volume of 10 μl. Each well was added with 2.5 μg erWalK protein, 10 nl 5,000 × Sypro Orange (Invitrogen) and different concentrations of small molecules. A HEPES buffer (100 mM HEPES, 150 mM NaCl, pH 7.5) was used to dilute the high-concentration protein stock of gel filtration-purified wild-type erWalK (in the buffer containing 100 mM NaCl, 10 mM Tris.HCl, pH7.5 and 1 mM DTT). Small molecules were added in nanolitre volume by a Labcyte Echo550 acoustic liquid transfer robot. Thermal scanning coupled with fluorescence detection was performed on a Bio-Rad real-time PCR machine CFX384. The fluorescence of the thermal transition was fitted to a Boltzmann function and normalized to the transition magnitude.

### Surface plasmon resonance experiment

To analyse the binding of DHBP to erWalK, SPR experiments were carried out using a Reichert SR7500DC SPR instrument (Reichert Technologies, Buffalo, NY). The binding assay was performed by using a Neutravidin Sensor Chip (Part #13206065) for high affinity capture of biotinylated erWalK. The biotinylation of erWalK was performed using the protocol described in (Technical Note 28, Biotinylation of protein for immobilization onto streptavidin biosensors, www.fortebio.com). The protein immobilization was at a flow rate of 33 μl min^−1^ in PBS for 3 min. For the analyte association, different concentrations of DHBP in PBS running buffer were injected for 3 min at a rate of 30 μl min^−1^ followed by a dissociation phase of 3 min. The sensor surface was regenerated after each dissociation cycle by allowing buffer to flow at 40 μl min^−1^ for a minimum of 15 min. Signals obtained for the erWalK bound surface were subtracted by signals obtained for the reference cell according to standard procedure using the system software. The concentration dependence of the subtracted signal was analysed to determine the binding affinity of the DHBP and erWalK interaction.

### Growth curve measurement

The Newman wild-type strain, D119A and V149A mutants were grown in TSB overnight. The cells were diluted into 200 μl fresh TSB with ∼2 × 10^5^ CFU with the supplementation of 75 μM DHBP (when indicated) and incubated at 37 °C for 24 h without shaking. The growth of the cells was monitored by measuring OD_600_ with the machine Bioscreen C (Growth Curves USA). The experiments were performed in triplicate.

### Size exclusion chromatography analysis

The proteins (after Ni-NTA purification) were concentrated to 2 ml and loaded into a gel-filtration column superdex 75 (GE Healthcare) for analysis in a gel filtration buffer (100 mM NaCl, 10 mM Tris.HCl, pH 7.5 and 1 mM DTT). The UV absorbance at 280 nm of the major peaks was normalized to a relative value 100.

## Additional information

**Accession codes:** The crystal structure of erWalKR86M was deposited in the RCSB Protein Data Bank (PDB) with PDB ID code: 4YWZ. The RNA-seq data were deposited in the National Center for Biotechnology Information Gene Expression Omnibus under series GSE75731.

**How to cite this article:** Ji, Q. *et al*. Structure and mechanism of the essential two-component signal transduction system WalKR in *Staphylococcus aureus*. *Nat. Commun.* 7:11000 doi: 10.1038/ncomms11000 (2016).

## Supplementary Material

Supplementary Information Supplementary Figures 1-8, Supplementary Tables 1-9 and Supplementary References.

## Figures and Tables

**Figure 1:** Structural characterization of erWalK reveals a canonical PAS domain. (**a**) The asymmetric unit of the crystal of erWalK contains an antiparallel homodimer. (**b**) Topology diagram of the structure of erWalK reveals a canonical PAS domain, as the β-strands are arranged in the order of 2-1-5-4-3. (**c**) Tertiary structure overlay of erWalK with a well-studied PAS domain protein DcuS PAS (PDB code: 3BY8) reveals four possible signal-transduction residues in erWalK. The structures of erWalK and DucS PAS are coloured pink and green, respectively; the ligand of DcuS PAS D-malate is coloured yellow. The potential signal-transduction residues of erWalK are indicated.

**Figure 2:** Mutation of the potential signal-transduction residues (D119A or V149A) impairs the function of WalKR TCS in *S. aureus*. (**a**) Mutation of D119 or V149 to Ala led to attenuated lysostaphin-induced lysis activity. Cells (WT/pCL55, D119A/pCL55, V149A/pCL55, D119A/p-*walKR* and V149A/p-*walKR*) were grown to OD_600_ of ∼1.6 before harvesting for analysis. The decline of OD_600_ was utilized to measure lysis activity. The experiments were performed in triplicate. (**b**) Almost fully abolished haemolysis activity was observed in the D119A and V149A mutants. (**c**) Mutation of D119 or V149 to Ala led to reduced biofilm production. The biofilm assay was performed in a polystyrene 96-well in TSB with the supplementation of 0.5% glucose and 3% NaCl. The experiments were performed in duplicate. (**d**) Mutation of D119 or V149 to Ala drastically reduced *S. aureus* survival in mice. Bacterial suspension (1 × 10^7^ CFU) was administered intravenously via retro-orbital injection into each of 10 6-week-old BALB/c mice. Colonization in liver and kidney was measured after 5 days of infection. Statistical analysis was performed using Student's *t*-test. Differences were considered statistically significant at *P* values<0.05. **P<0.01; *P<0.05. The experiments were performed in duplicate. The error bars represent the s.d. of the analysed data.

**Figure 3:** Transmission electron microscopy test showed mutation of the potential signal-transduction residue (D119A) resulted in defective cell morphology. Cells were grown to OD_600_ of ∼0.6 before harvesting for analysis. Scale bars, 200 nm.

**Figure 4:** Broad transcription changes were observed in the D119A and V149A mutants. (**a**) Venn diagram of the number of genes whose expressions are downregulated in the D119A mutant overlapping genes whose expressions are downregulated in the V149A mutant as compared with the wild-type strain. ‘−': genes whose expressions are downregulated. (**b**) Grouping genes that are differentially expressed in the D119A mutant compared with the wild-type strain indicated in the diverse roles of WalKR TCS. (**c**) The majority of downregulated genes are involved in cell wall metabolism, pathogenesis and regulation in the D119A mutant, which is consistent with genes whose expressions were upregulated in the WalRD55E mutant as compared with the wild-type strain.*: genes that exist in both lists. Black bars represent genes that are absent in the transcriptional profiling list of the V149A mutant, while red bars represent genes that are present in the transcriptional profiling list of the V149A mutant.

**Figure 5:** DHBP is capable of activating WalKR TCS via targeting erWalK. (**a**) Thermal shift assay indicates the direct binding of DHBP to erWalK. (**b**) DHBP selectively promotes the lysostaphin-induced lysis activity of the Newman wild-type strain, but not the D119A mutant. Cells were grown to OD_600_ of ∼1.4 with the supplementation of 75 μM DHBP (as indicated) before harvesting for analysis. The decline of OD_600_ was utilized to measure lysis activity. The experiments were performed in triplicate. The error bars represent the s.d. of the analysed data.

**Figure 6:** DHBP treatment triggers profound transcription changes in *S. aureus*. (**a**) Venn diagram of the number of genes whose expressions are upregulated upon DHBP treatment overlapping genes whose expressions are downregulated in the D119A mutant as compared with the wild-type strain. −: genes whose expressions are downregulated; and +: genes whose expressions are upregulated. (**b**) The majority of upregulated genes upon DHBP treatment are involved in cell wall metabolism and pathogenesis, which is consistent with genes whose expressions are downregulated in the D119A mutant as compared with the wild-type strain. *: genes that exist in both lists.

**Table 1:** Data collection, phasing and refinement statistics.

	**erWalK6R86M (seleno-Met)**
*Data collection and crystal parameters*	
Space group	P32
Wavelength (Å)	0.97856
	
*Cell dimensions*	
a, b, c (Å)	66.701, 66.701, 80.492
α, β, γ (°)	90.000, 90.000, 120.000
Resolution (Å)	30.00–1.70
*R*_merge_ (%)	5.9 (65.0)*
*I/σI*	41.4 (3.1)
Completeness (%)	100 (100)
Redundancy	5.7 (5.7)
	
*Refinement*	
Reflections (#)	44,089
*R*_work_/*R*_free_ (%)	17.9/21.2
	
*Number of non-hydrogen atoms (#)*	
Protein	2,364
Water	386
	
*r.m.s.d.*	
Bond lengths (Å)	0.013
Bond angle (°)	1.533
	
*Average B factors* (Å^2^)	
Overall	31.2
Protein	29.5
Water	42.0

^*^Numbers in parentheses represent statistics in highest-resolution shell.
